# 6,12-Diphenyl-3, 9-diazatetraasterane-1, 5, 7, 11-tetracarboxylate Inhibits Proliferation, Migration and Promotes Apoptosis in Ovarian Cancer Cells

This article has been retracted.

**DOI:** 10.1155/2020/5068067

**Published:** 2020-09-03

**Authors:** Pingping Chen, Huibing Wang, Meng Li, Linqi Yang, Feifei Mou, Bhupinder Singh, Jing-Yu He, Wei Zhang

**Affiliations:** ^1^Department of Pharmacology, College of Basic Medicine, Hebei University of Chinese Medicine, Shijiazhuang, 050200 Hebei Province, China; ^2^Department of Nursing, Shijiazhuang Medical College, Shijiazhuang, 050500 Hebei Province, China; ^3^College of Basic Medicine, Hebei Medical University, Shijiazhuang, 050017 Hebei Province, China; ^4^College of Chemical Engineering, Shijiazhuang University, Shijiazhuang, 050035 Hebei Province, China

## Abstract

6,12-Diphenyl-3,9-diazatetraasterane-1, 5, 7, 11-tetracarboxylate (DDTC) has been synthesized by the photodimerization of 4-phenyl-1,4-dihydropyridine-3,5-dicarboxylate. The potential of theercvantitumor activity and mechanism were investigated *in vitro* using MTT assay in human lung cancer cell line A549, ovarian cancer cell lines SKOV3 and A2780, breast cancer cell line MCF-7, gastric cancer cell line BGC-823, colon cancer cell line HT29, prostate cancer cell line DU145, and liver cancer cell line SMMC7721. The results show that DDTC can inhibit the growth of ovarian cancer SKOV3 and A2780 cells. The best IC_50_ value is approximately 5.29 ± 0.38 and 4.29 ± 0.39 *μ*M, respectively. DDTC induced the cell cycle arrest in the G2 phase by flow cytometric analysis. The migration and invasion of ovarian cancer SKOV3 and A2780 cells were inhibited by DDTC. DDTC could increase the expression protein level of E-cadherin in A2780 cells and ascend the expression protein and mRNA levels of E-cadherin in SKOV3 cells. DDTC could also decrease the protein and mRNA expression of EMT (epithelial-to-mesenchymal transition) markers of N-cadherin and Vimentin. mRNA and protein expression level of checkpoint kinase 1 (Chk1) were significantly increased and expressions of cyclin-dependent kinase (CDK1) and cell division cycle 25a (Cdc25a) were decreased in the SKOV3 and A2780 cell lines. Moreover, DDTC induced apoptosis by the cleavage and activation of caspase 3 and caspase 9.

## 1. Introduction

The structure of 6,12-diaryl-3,9-diazatetraasterane-1,5,7,11-tetracarboxylates (Figure 1) has been synthesized as a therapeutic agent for inhibiting the activity of the HIV-1 protease [1, 2]. However, the antitumor effect of 3,9-diazatetraasterane(DDTC) on cancer and the underlying mechanisms remain unknown. We synthesized with DDTC to investigate the influence on the antitumor activities and the effects of DDTC on proliferation and apoptosis of human carcinoma cells.

## 2. Materials and Methods

### 2.1. Reagents and Chemicals

Fetal bovine serum (FBS) was obtained from HyClone (USA), and RPMI (Roswell Park Memorial Institute) 1640 medium, DMEM (Dulbecco's Modified Eagle Medium), penicillin, streptomycin, and all other reagents were obtained from Gibco (USA). DDTC, synthesized by the College of Chemical Engineering, Shijiazhuang University, was dissolved in DMSO and the final concentration of DMSO in cultures was ≤0.1%(*v*/*v*).

### 2.2. Cell Culture

The human lung cancer cell line A549, human breast cancer cell line MCF-7, human gastric cancer cell line BGC-823, ovarian cancer cell lines SKOV3 and A2780, human liver cancer cell line SMMC-7721, colon cancer HT29 cells, and prostate cancer DU145 cells were cultured in RPMI1640 medium with 10% (*v*/*v*) FBS and penicillin (100 U/ml)/streptomycin (100 mg/ml) at 37°C in the moisture-saturated atmosphere containing 5% CO_2_.

### 2.3. Antiproliferative Activity Assay

Briefly, human lung cancer A549 cells, ovarian cancer SKOV3 and A2780 cells, breast cancer MCF-7 cells, gastric cancer BGC-823 cells, colon cancer HT29 cells, prostate cancer DU145 cells, and liver cancer SMMC7721 cells were seeded into 96-well plates for 24, 48, and 72 hours at 37°C, respectively. An antiproliferation assay was performed by the MTT method. [3] Tests were repeated three times.

### 2.4. Migration and Invasion Assay

SKOV3 and A2780 cells were cultured in RPMI1640 medium with 2% serum accompanied with 0.1, 1, and 10 *μ*M DDTC for 48 h. The capacity of migration was cleared via a pipette tip (10 ml) for wound healing assay. The superculture chamber (Corning, USA) with BD Matrigel Matrix (BD Biosciences, NY, USA) was employed for Transwell assay. The cells were stained with 0.5% methylrosaniline chloride (Sigma Aldrich), evaluated by the digital medical image analysis system (Leica DM2500, Germany) and light microscope (Leica DMIL-PH1, Germany).

### 2.5. Flow Cytometry Assay

SKOV3 and A2780 cells were exposed to 0.1, 1, and 10 *μ*M DDTC for 48 h. The cells were harvested (trypsinization and centrifugation) and fixed with 75% ethanol. Next, 50 *μ*g/ml propidium iodide in a phosphate-citrate buffer (pH 7.2) was incubated. Cellular DNA content was determined through flow cytometry using FACSCalibur system (BD Biosciences, Franklin Lakes, New Jersey, USA) for cell cycle progression assessment.

### 2.6. Western Blot Assay

SKOV3 and A2780 cells were treated with DDTC at 0.1, 1, and 10 *μ*M for 48 h. After three times washing with PBS, the cells were lysed for 30 min on ice and centrifuged at 10000×g for 5 min at 4°C. The contents of segregated proteins in cell lysates were quantified using an ND-1000 Spectrophotometer (NanoDrop, Wilmington, Delaware, USA). Equal amounts of protein samples were segregated through 10% SDS-PAGE (polyacrylamide gel electrophoresis) and transferred onto PVDF membranes (Millipore, Bedford, Massachusetts, USA). After 5% milk block for 2 h, immunoblotting was done with primary antibodies overnight at 4°C. The primary antibodies include Cdc25a (AF6252, at 1 : 300 dilution), CDK1 (ET1605-54, at 1 : 300 dilution), Chk1 (ET1609-71, at 1 : 300 dilution), Vimentin (ab92547, at 1 : 3000 dilution), N-cadherin (AF4039, at 1 : 500 dilution), E-cadherin (AF0131, at 1 : 500 dilution), caspase 3 (ET1602-39, at 1: 500 dilution), caspase 9 (AF6348, at 1 : 500 dilution), cleaved caspase 3 (AF7022, at 1 : 500 dilution), cleaved caspase 9 (AF5240, at 1 : 500 dilution), and *β*-actin (AC026, at 1 : 10000 dilution). Next, the membranes were incubated with secondary antibodies of goat anti-rabbit IG (KPL074-1506, at 1 : 5000 dilution) for 1 h at 37°C. The intensity of protein bands was estimated via executing Fusion FX5 Spectra (Fusion, France).

### 2.7. Real-Time Fluoresce Quantitative PCR (Q-PCR)

According to the manufacturer's instruction (Nippon Gene Co. Ltd., Tokyo, Japan), the total RNA was procured from the SKOV3 and A2780 cells, which were treated with DDTC for 48 hours. After spectrophotometric quantification at 260 nm, total RNA (1 mg) was converted into cDNA by Reverse Aid First-Strand cDNA Synthesis kit (Thermal Scientific Co. Ltd., USA). Using the reaction mixtures (20 *μ*l) by the Real-Time PCR system (BIOER Co. Ltd., Japan) containing cDNA, primer pairs (Table 1), and platinum SYBR Green Q-PCR Super Mix-UDG (Invitrogen, Life Technologies Co. Ltd., USA). The relative gene expressions were calculated using2^-*ΔΔ*Ct^ method, as described previously. [3]

## 3. Results

### 3.1. Antiproliferative Activity of DDTC

The antiproliferative activity of DDTC was assessed in human lung cancer cells A549, ovarian cancer cells SKOV3 and A2780, breast cancer cells MCF-7, gastric cancer cells BGC-823, colon cancer cells HT29, prostate cancer cells DU145, and liver cancer cells SMMC7721 *in vitro*.  Table 2 shows the IC_50_ of DDTC on different cancer cell lines for 24 h, 48 h, and 72 h, respectively. As a result, the effects of DDTC on the growth of SKOV3 and A2780 cells for 48 h were stronger than those on A549, HT29, MCF-7, BGC-823, DU145, and SMMC7721 cells (Table 2). So, we selected SKOV3 and A2780 cell lines to conduct subsequent experiments.

### 3.2. Effect of DDTC on Migration in Ovarian Cancer Cells

The wound healing and Transwell assay were performed to explore the DDTC mechanistic study in ovarian cancer cell lines. The significant different results were showed that the compound of DDTC inhibited migration in ovarian cancer SKOV3 and A2780 cells, respectively (Figure 2).

### 3.3. Effect of DDTC on EMT Markers in Ovarian Cancer Cells

EMT is a key factor of epithelial carcinoma dissemination which includes cancer migration, invasion, and transport through the blood/lymph vessels in tumors. [4] Many signal pathways are involved in the EMT progression, such as Wnt/*β*-catenin, TGF, MMPs, and Notch signaling pathways. [5] The result indicated that DDTC could regulate the expression protein level of E-cadherin and downregulate the expression protein and mRNA levels of N-cadherin and Vimentin in A2780 and SKVO3 cells, as well as upregulate the expression mRNA level of E-cadherin in A2780 cells (Figure 3).

### 3.4. Effect of DDTC on Cell Cycle Progression

The proliferation of cells is closely related to the cell cycle. The results of the MTT assay provided the first evidence of the antiproliferative effect of DDTC, so we used flow cytometric analysis to evaluate whether DDTC induces the cell cycle arrest. According to the results of flow cytometric analysis, DDTC increased the cell population at the G2 phase in SKOV3 and A2780 cells (Figure 4).

### 3.5. Effects of DDTC on Cell Cycle Regulators

Chk1, Cdc25a, and CDK1 were proved to be linked to cell cycle arrest, which could regulate cell proliferation. CDKs control cell progression by binding with cyclins. Cyclin B1 induces cell cycle G2 to the M phase by activation of CDK1. Cdc25a is an important regulator in cell proliferation. Chk1 leads to DNA damage by inhibiting Cdc25a activity [6, 7]. As shown in Figure 5, the expression of CDK1, Chk1, and Cdc25a proteins and mRNA by Western blot and Q-PCR indicated that DDTC could reduce the expression of Cdc25a and CDK1 and increase of Chk1, which is consistent with the G2 arrest induced by DDTC.

### 3.6. Effects of DDTC on Apoptosis-Relevant Proteins

Apoptosis is a genetically regulated process of cell suicide, which is modulated by a variety of cellular signaling pathways. The central component of the apoptotic machinery is a proteolytic system consisting of caspases [8]. Therefore, we used western blotting and Q-PCR to analyze the mechanisms of DDTC-induced apoptosis. The effect of DDTC treatment on the expression of caspases 3 and -9 and cleaved caspases 3 and 9 were also examined. DDTC reduced the expression of caspase 3 and 9 proteins and mRNA, but increased the expression of the cleaved caspase 3 and 9 proteins and mRNA (Figure 6).

## 4. Discussion

In this study, we have provided evidence of the antitumor effect of DDTC. Firstly, we selected several human cancer cells lines including lung cancer cell line A549, ovarian cancer cell lines SKOV-3 and A2780, breast cancer cell line MCF-7, gastric cancer cell line BGC-823, colon cancer cell line HT29, prostate cancer cell lines DU145, and liver cancer cell line SMMC-7721 to confirm whether DDTC could inhibit the growth of cancer cells. According to the results of the MTT assay, the inhibitory effect of DDTC on the proliferation of ovarian cancer was more effective than that on the other cancers mentioned above.

Therefore, we study the anticancer mechanism of DDTC further.

The migration of cancer cells is closely related to the proliferation of cells, so we used the wound healing and Transwell assay to detect the effect of DDTC on the migration and invasion. These confirmed that DDTC inhibited migration were consistent with increasing the protein expression levels of E-cadherin and decreasing the protein and mRNA expression levels of EMT markers (N-cadherin and Vimentin) in ovarian cancer cells.

MTT assay result provided the first evidence of the antiproliferative effect of DDTC. Flow cytometric analysis showed that DDTC induced cell cycle arrest at the G2 phase in A2780 and SKOV3 cells. CDK1 is a key regulator of the cell cycle at this checkpoint. The activation of CDK1 is critical to the cell cycle of the transition from the G2 to M phase. [3, 6] Chk1 inhibits the Cdc25a activity meanwhile Cdc25a promotes activation of CDK1 [7, 8]. Our result demonstrated that DDTC reduced the expression level of Cdc25a and CDK1 and increased Chk1 expression.

Checkpoints induce cell cycle arrest, which closely links to cell DNA damage and apoptosis. Apoptosis was proved regulated by many cellular pathways and decrease the activities of caspase 3 and caspase 9, which was related to the tumor development [9, 10]. In our study, Q-PCR and western blot were used to analyze the mechanisms of DDTC-induced apoptosis. DDTC increased the protein and mRNA levels of cleaved caspase 9 and caspase 3, and reduced the expression of caspase 9 and caspase 3 genes and proteins in the SKOV3 and A2780 cells, which indicated that DDTC-induced apoptosis by cleavage and activation of caspases.

## 5. Conclusion

In summary, DDTC could inhibit the growth of human cancer cells and display remarkable antitumorigenic activities, which included the effect of DDTC on the cell cycle checkpoints, migration and invasion in ovarian cancer cells. The DDTC exhibited an ability to increase the expression of cleaved caspase 9 and cleaved caspase 3 proteins and reduced the expression of caspase 9 and caspase 3 proteins in SKOV3 and A2780 cells, which indicated that DDTC induced apoptosis by the caspase-dependent pathway. All these results illustrated that DDTC could be a potential drug candidate to treat ovarian cancer.

## Figures and Tables

**Figure 1:** The structure of DDTC.

**Figure 2:** The effect of DDTC on the invasion and migration in ovarian cancer cells. The dosage of DDTC at 0.1 *μ*M, 1 *μ*M, and 10 *μ*M in SKOV3 and A2780 cells. (a) DDTC inhibited the invasion in SKOV3 cells. (b) DDTC inhibited the invasion in A2780 cells. (c) DDTC inhibited the migration in SKOV3 cells. (d) DDTC inhibited the migration in A2780 cells.

**Figure 3:** The effect of DDTC on the EMT in ovarian cancer cells. The dosage of DDTC at 0.1 *μ*M, 1 *μ*M, and 10 *μ*M in SKOV3 and A2780 cells. (a, b) DDTC increased the protein expression level of E-cadherin and decreased the protein expression level of N-cadherin and Vimentin in SKOV3 cells. (c, d) DDTC increased the protein expression level of E-cadherin and decreased the protein expression level of N-cadherin and Vimentin in A2780 cells. (e) DDTC decreased the mRNA expression level of N-cadherin and Vimentin in SKOV3 cells. (f) DDTC increased the mRNA expression level of E-cadherin and decreased the mRNA expression level of N-cadherin and Vimentin in A2780 cells.

**Figure 4:** Analysis of cell cycle progression by flow cytometry. The dosage of DDTC at 0.1 *μ*M, 1 *μ*M, and 10 *μ*M in SKOV3 and A2780 cells. (a, c) DDTC increased cell population at the G2 phase of SKOV3 cells. (b, d) DDTC increased cell population at the G2 phase of A2780cells.

**Figure 5:** The effect of DDTC on expression of cell cycle regulators. The dosage of DDTC at 0.1 *μ*M, 1 *μ*M, and 10 *μ*M in SKOV3 and A2780 cells. (a, b) Western blot assay showed that DDTC upregulated the expression of Chk1 protein level and downregulated the expression of Cdc25a and CDK1protein levels in SKOV3 cells. (c, d) Western blot assay showed that DDTC upregulated the expression of Chk1 protein level and downregulated the expression of Cdc25a and CDK1protein levels in A2780 cells. (e) The mRNA level of Chk1 was increased and level of Cdc25a and CDK1 were decreased in SKOV3 cells by Q-PCR. (f) The mRNA level of Chk1 was increased and level of Cdc25a and CDK1 were decreased in A2780 cells by Q-PCR. ^∗^*P* < 0.05; ^∗∗^*P* < 0.01 vs. the control group.

**Figure 6:** The effect of DDTC on the expression of caspase 3, cleaved caspase 3, caspase 9, and cleaved caspase 9. The dosage of DDTC at 0.1 *μ*M, 1 *μ*M, and 10 *μ*M in SKOV3 and A2780 cells. (a, b) Western blot assay showed that DDTC downregulated the expression of caspase 3 and caspase 9 protein levels and upregulated the expression of cleaved caspase 3 and cleaved caspase 9 protein levels in SKOV3 cells andA2780 cells. (c, d) Western blot assay showed that DDTC downregulated the expression of caspase 3 and caspase 9 protein levels and upregulated the expression of cleaved caspase 3 and cleaved caspase 9 protein levels in A2780 cells. (e) The mRNA levels of caspase 3 and caspase 9 were decreased, and levels of cleaved caspase 3 and cleaved caspase 9 were increased in SKOV3 cells by Q-PCR. (f) The mRNA levels of caspase 3 and caspase 9 were decreased and levels of cleaved caspase 3 and cleaved caspase 9 were increased in A2780 cells by Q-PCR. ^∗^*P* < 0.05; ^∗∗^*P* < 0.01 vs. the control group.

**Table 1:** The sequences of 8 pairs of primers.

Primers	Forward (5′-3′)	Reverse (5′-3′)
Chk1	CTCCTCAGCATCTTATCCGAGT	GCTGTTCCGTCCCAGTAGATTA
Cdc25a	CTGGATAATGGTGAATGGACAC	CGATGTGGCATACTTGTTCTTG
CDK1	CTGGACACTGAGAGGGCAATC	AAATGGGAAGGAGAAGGAGAAG
Caspase 3	ATGGAGAACAATAAAACCT	CTAGTGATAAAAGTAGAGTTC
Cleaved caspase3	CCATAAAAGCACTGGAATGTCA	CCGTTCGTTCCAAAAATTACTC
Caspase 9	GGCTGTCTACGGCACAGATGGA	CTGGCTCGGGGTTACTGCCAG
Cleaved caspase9	AAACTGTCCAGCACTTTCA	GGTCCCGTAAAGCAACAT
Vimentin	TGCCGTTGAAGCTGCTAACTA	CCAGAGGGAGTGAATCCAGATTA
N-cadherin	TTTGATGGAGGTCTCCTAACACC	ACGTTTAACACGTTGGAAATGTG
E-cadherin	AAAGGCCCATTTCCTAAAAACCT	TGCGTTCTCTATCCAGAGGCT
*β*-Actin	TGACGTGGACATCCGCAAAG	CTGGAAGGTGGACAGCGAGG

**Table 2:** IC_50_ of DDTC on different cancer cell lines.

TTime (hour)	IC50 (*μ*M) (mean ± SD)							
	A549	SKOV3	A2780	MCF-7	BGC-823	HT29	DU145	SMMC7721
24	89.24 ± 8.98	65.29 ± 6.89	74.29 ± 7.39	>100	>100	>100	>100	>100
48	8.59 ± 0.46	5.29 ± 0.38	4.29 ± 0.39	20.01 ± 0.56	>100	>100	>100	>100
72	7.88 ± 0.37	4.19 ± 0.27	3.99 ± 0.41	18.12 ± 0.66	>100	>100	>100	>100

## Data Availability

The data are available upon direct request to the corresponding author.
